The article "Rapid Detection of vanA Resistance Gene from E. faecalis Clinical Isolates Using Duplex Loop-Mediated Isothermal Amplification and Triplex PCR Assay" was published in 2022. Journal: Biomed Res Int.

# Rapid Detection of *vanA* Resistance Gene from *E. faecalis* Clinical Isolates Using Duplex Loop-Mediated Isothermal Amplification and Triplex PCR Assay

**DOI:** 10.1155/2022/4384196

**Published:** 2022-09-20

**Authors:** Mohsen Azizi, Hamid Motamedi, Hadi Hossainpour, Ramin Abiri, Mahsa Kashef, Kamal Ahmadi, Jale Moradi, Amirhooshang Alvandi

**Affiliations:** ^1^Department of Microbiology, School of Medicine, Kermanshah University of Medical Sciences, Kermanshah, Iran; ^2^Student Research Committee, School of Medicine, Kermanshah University of Medical Sciences, Kermanshah, Iran; ^3^Fertility and Infertility Research Center, Health Technology Institute, Kermanshah University of Medical Sciences, Kermanshah, Iran; ^4^Medical Technology Research Center, Health Technology Institute, Kermanshah University of Medical Sciences, Kermanshah, Iran

## Abstract

Today, the spread of vancomycin-resistant strains isolated from *Enterococcus faecalis* (*E. faecalis*) has become a major health concern worldwide. Therefore, it is essential to provide a rapid and sensitive assay for identifying *vanA* gene for timely and appropriate antimicrobial control of resistant enterococcal infections. For this purpose, a cross-sectional study was performed on different clinical specimens of enterococci from Imam Reza hospital, Kermanshah, Iran. The antimicrobial susceptibility testing was determined by disk diffusion and MIC methods. Triplex-PCR and duplex-LAMP assays were also used to identify *vanA E. faecalis* resistance gene isolates. The results of this study shown that out of 108 *Enterococcus* isolates, 86, 18, 2, 1, and one isolates of *E. faecalis*, *E. faecium*, *E. avium*, *E. psudoavium*, and *E. raffinosus* were identified, respectively. On the other hand, *E. faecalis* was confirmed in 87 and 88 isolates using duplex-LAMP and triplex PCR, respectively. The LAMP primer set designed in this study can reliably identify seven distinct regions of the *vanA* gene, and finally the sensitivity, specificity, and the positive and negative predictive values of LAMP assay were shown to be 94.19%, 72.73%, 76.19%, and 93.10%, respectively. In general, sample processing, isothermal reaction and result reporting were completed using the LAMP assay in 75 minutes. Our findings suggest that LAMP assay has been approved as an alternative to the vancomycin resistance *Enterococcus* genotype (*vanA* and *vanB*) compared to other methods and has the advantage of being rapid, time-consuming, and easy for diagnosis.

## 1. Introduction

Enterococci are positive gram cocci that are ubiquitous in the gastrointestinal tract of animals and humans, and even in water and soil [1]. However, this organism recognized as predominantly nonpathogenic bacteria is sometimes opportunistic and causes human diseases [2]. *E. faecium* and *E. faecalis* are two common species of enterococci that are now recognized as the most important hospital-acquired infections such as bacteremia and urinary tract infections [3, 4]. In the 1970s and 1980s, *E. faecium* first developed high levels of resistance to ampicillin and during the 1980s became resistant to aminoglycosides, fluoroquinolones, and glycopeptides, especially vancomycin [5–7]. On the other hand, *E. faecalis* is resistant to aminoglycosides, but resistance to ampicillin and vancomycin is infrequent than *E. faecium* [8]. Vancomycin was previously considered the “last line of treatment” for the treatment of severe infections caused by multidrug-resistant enterococci [9]. Acquired resistance to vancomycin is caused by 37 different clusters (*vanA*, *B*, *D*, *E*, *F*, *G*, *L*, *M*, and *N*) of which *vanA* is clinically significant [3]. In addition, the plasticity of enterococcal genomes by the *vanA* gene allows the organism to respond rapidly and with limitations by obtaining genetic determinants that enhance its ability to colonize or infect the host [10]. Conventional diagnosis of vancomycin resistance by culture-based methods (Kirby-Bauer and broth dilution) is both require an experienced laboratory expert and time-consuming. On the other hand, molecular detection techniques (such as conventional and real-time PCR methods) require specialized and expensive tools and consumables. Therefore, it is important to have a rapid, sensitive, and cost-effective assay for identifying vancomycin resistance genes. For this reason, in recent years, loop-mediated isothermal amplification (LAMP) assay has been considered for the detection of vancomycin resistance genes due to its specificity and high sensitivity [11]. LAMP requires only a temperature-controlled water- or dry-bath, and the results can be analyzed directly by the naked eye [12]. The focus of this study is LAMP assay for rapid and sensitive detection of the *vanA* gene in *Enterococcus* species isolated from different clinical specimens.

The article "Rapid Detection of vanA Resistance Gene from E. faecalis Clinical Isolates Using Duplex Loop-Mediated Isothermal Amplification and Triplex PCR Assay" was published in 2022. Journal: Biomed Res Int.

## 2. Materials and Methods

### 2.1. Bacterial Strains

A total of 108 *Enterococcus* strains were collected from different clinical specimens including blood, urine, wound, and CSF from Imam Reza Hospital in Kermanshah, Iran. Then, bile esculin agar, sodium azide selective medium, blood agar (Merck, Germany) and also API 20 Strep (bioMerieux, France) were used to detect *Enterococcus* strains. Biochemical tests such as catalase, growth in 6.5% NaCl, arabinose, pyruvate, and sorbitol fermentation were also used to differentiate *Enterococcus* strains [13]. These strains were stored in 10% glycerol broth (w/v) at − 70 °C for later steps. This study was ethically approved by the Kermanshah University of Medical Sciences, Institutional Review Board (IR. KUMS.REC.1394.498).

### 2.2. Disk Diffusion and MIC Methods

Two methods of disk diffusion and Minimum Inhibitory Concentration (MIC) were used to test the antimicrobial susceptibility of *E. faecalis* and *E. faecium* isolates. Antibiotic susceptibility testing was carried out using Kirby-Bauer disk diffusion method according to the Clinical and Laboratory Standard Institute (CLSI) guidelines [14]. Antibiotics used (Mast, England) included ampicillin (10 micrograms), penicillin (10 micrograms), ciprofloxacillin (5 micrograms), norfloxacin (10 micrograms), and erythromycin (15 micrograms). Broth microdilution method was used for vancomycin susceptibility testing according to CLSI guidelines, with a range of 0.0625 to 64 micrograms/mL. Vancomycin resistant breakpoint was considered equal or more than 32 micrograms/mL [15].

### 2.3. Genomic DNA Preparation

The genomic DNA templates were extracted from all culture strains using DNA extraction kits AccuPrep® Genomic DNA extraction kit (Bioneer, South Korea) according to the manufacturer's instructions. The extracted templates were tested with ultraviolet spectrophotometer (Nano drop Technologies, Inc., Wilmington, DE, USA) at A260/280. On the other hand, the templates were stored under at − 20 °C before the templates were used.

### 2.4. PCR and LAMP Primer Design

For detection of *Enterococcus* genus, six pairs of the LAMP primers for each target (*vanA* and *E. faecalis* species) were separately designed using primer explorer software version 4 (http://primerexplorer.jp/e/). More than 1000 sets of the primers screened to select two of them that can develop different pattern when compared together. There were four primers needed for PCR reaction; to design these primers, the whole genome of *E. faecalis* and *E. faecium* has been downloaded from NCBI gene bank; then, the primers were designed with consideration of multiplex-PCR. Primers for LAMP assay have been designed with primer explorer software version4. All the primers are listed in Table 1.

### 2.5. PCR Assay

The reaction mixture for multiplex-PCR assay was 25 *μ*L that was prepared as follows: 12.5 *μ*l of 2× Taq premix Master mix (Ampliqon UK), 7.5 *μ*l of sterile double distilled water, 1 *μ*l of each forward and reverse primer, and 3 *μ*l of DNA sample. The DNA samples as well as a quality control (*E. faecalis* strain ATCC 29212) was amplified for *vanA* gene by an initial denaturation step for 5 min at 95 °C followed by 35 cycles of 92 °C for 30 s, 55 °C for 30 s, and 72 °C for 1 min and a final extension step at 72 °C for 5 min in a Bio-Rad Thermal Cycler (Bio-Rad Laboratories, Inc., USA).

The article "Rapid Detection of vanA Resistance Gene from E. faecalis Clinical Isolates Using Duplex Loop-Mediated Isothermal Amplification and Triplex PCR Assay" was published in 2022. Journal: Biomed Res Int.

### 2.6. LAMP Reaction

LAMP reaction was carried out in a final volume of 45 *μ*l containing 1.6 mM each of FIP and BIP, 0.2 mM each of B3 and F3, 0.8 mM each of LB and LF, 2 *μ*M dNTP, 0.8 M betaine, 1.5× buffer,12 mM MgSO_4_, and 3 *μ*l target DNA. LAMP reactions were incubated in a program as follows: initial denaturation 92 °C for 3 min; after adding 8 U Bst polymerase, reaction continued with amplification at 65 °C for 60 min and end of amplification in at 92 °C for 1 min. In addition to a positive control, a negative control was included to monitor for possible cross-contamination.

### 2.7. Analytical Sensitivity and Specificity of LAMP and Multiplex-PCR

The specificity of the each duplex-LAMP and multiplex-PCR methods were determined using performing reaction on purified DNA of some bacteria including *E. faecium*, *E. avium*, *E. raffinosus*, *E. psudoavium*, *E. hirae*, *E. durans*, *streptococcus pneumonia*, and *staphylococcus aureus*. All species were confirmed using standard biochemical tests. To determine the LAMP limit of detection (LOD) for *E. faecalis*, a fresh suspension of *E. faecalis* reference strain broth culture has been prepared in Mueller Hinton Agar (MHA) to reach the concentration of 4 McFarland (12 × 10^8^) CFU/ml. The DNA of suspension was extracted using specific kit and the concentration of DNA of that measured using NanoDrop (Thermo Fisher Scientific, USA). Then, ten-fold serial dilutions of purified DNA were prepared, and 3 *μ*l of each diluted DNA was used as DNA template for PCR and LAMP assay [16]. For the construction of a multiplex LAMP (mLAMP), we modified the FIPs and BIPs by inserting a restriction enzyme (*EcoRI*) cleavage site between the F1 complementary and F2 and between the B1 complementary and B2, respectively, as shown in Table 1. To confirm the LAMP amplification product specificity, restriction fragment length polymorphism (RFLP) analysis was performed with the restriction enzyme *EcoRI* (Jena Bioscience, Germany). The specific restriction sites in the LAMP products were analyzed and selected with NEB cutter V2.0 (http://toolshttp://neb.com/NEBcutter2). Briefly, the DNA products amplified by LAMP were digested with 1.5 U/*μ*l *EcoRI* following the manufacturer's standard protocol. *EcoRI* can specifically digest the DNA sequence 5′-GAATTC-3′. The final digestion products were expected to be 170 and 135 bases [17].

### 2.8. Spiked Blood Culture Specimens

Spiked blood culture was prepared to evaluate the ability of LAMP to detect organism in clinical specimens. Starting with a 1-McFarland standard suspension of organism, three successive 100-fold dilutions were performed by placing 10 *μ*l of suspension into 990 *μ*l of diluent. This was followed by a 30-fold dilution through placement of 100 *μ*l of suspension into a blood culture bottle with 3 ml of banked blood, to produce a final organism concentration between 10 and 100 CFU/ml. Colony counts were performed prior to the final 1 : 30 dilution, to verify the organism concentration [16].

The article "Rapid Detection of vanA Resistance Gene from E. faecalis Clinical Isolates Using Duplex Loop-Mediated Isothermal Amplification and Triplex PCR Assay" was published in 2022. Journal: Biomed Res Int.

### 2.9. Detection of Amplified Product

Amplified product in single LAMP reaction was analyzed using naked eye for detection of pyrophosphate sediment. For detection of amplification in duplex-LAMP, one *μ*L of the LAMP product or *EcoRI* digested products were subjected to 1.5% agarose gel electrophoresis and visualized using transilluminator. For detection of specific PCR amplification, 5 *μ*l of PCR product was subjected to electrophoresis through 1.5% agarose gel, stained with ethidium bromide, and visualized using transilluminator.

### 2.10. Statistical Analysis

The analysis was performed using the SPSS version 19 (Chicago, IL, USA). Data were analyzed using the chi-square test and Fisher's exact test, with significance set at *p* value < 0.05. Diagnostic test value of each test was calculated using MedCalc's online software.

## 3. Results

### 3.1. Enterococci Isolates

Among 108 clinical samples, 86 isolates (79.62%) were identified *E. faecalis*, 18 isolates *E. faecium* (16.66%), two isolates *E. avium* (1.85%), one isolate *E. psudoavium* (0.91), and also one isolate *E. raffinosus* (0.91) using culture method. The results of the collected samples are shown in Table 2.

### 3.2. Antimicrobial Susceptibility Testing

The rate of resistance to ampicillin, penicillin, gentamicin, erythromycin, and ciprofloxacin norfloxacin, among *E. faecium* isolates, was 91.66%, 83.33%, 75%, 83.33%, 66.66%, and 58.33%, respectively. Meanwhile, *E. faecalis* isolates exhibited 5.81%, 5.81%, 33.72%, 54.65%, 40.69%, and 34.88% resistance to ampicillin, penicillin gentamicin, erythromycin, ciprofloxacin, and norfloxacin, respectively. The results of microdilution method showed that 8 isolates were phenotypically resistant to vancomycin.

### 3.3. Clinical Specificity and Sensitivity of the LAMP Assay

Sensitivity, specificity, positive predicting value (PPV), and negative predicting value (NPV) of the duplex-LAMP and PCR in comparison with gold standards culture were as the same 94.19%, 72.73%, 76.19%, and 93.10%, respectively. There was perfect agreement between lamp and culture as gold standard methods with kappa coefficient of %8981. While kappa coefficient for PCR and API were %8981 and %8333, respectively. The results are shown in Table 3.

The article "Rapid Detection of vanA Resistance Gene from E. faecalis Clinical Isolates Using Duplex Loop-Mediated Isothermal Amplification and Triplex PCR Assay" was published in 2022. Journal: Biomed Res Int.

### 3.4. Analytical Specificity of the Primers

To evaluate the analytical specificity of the primer sets, single and multiplex-PCR and also single and duplex-LAMP were carried out on purified extracted DNA from *E. faecium*, *E. avium*, *E. raffinosus*, *E. psudoavium*, *E. hirae*, *E. durans*, *Streptococcus pneumoniae*, and *Staphylococcus aureus*. All species were fully identified using standard biochemical tests. The results were shown that single and duplex-LAMP and PCR only were positive for *E. faecalis* are shown in Figures 1 and 2.

### 3.5. Analytical Sensitivity (LOD)

The detection limits of duplex-LAMP and multiplex-PCR were determined using 10-fold serial dilutions of *E. faecalis* DNA. The LOD for multiplex-PCR was 1 pg/reaction and for duplex-LAMP reaction was 10 fg/reaction. It means that the analytical sensitivity of the duplex-LAMP was 100-fold more sensitive than multiplex-PCR that is shown in Figure 3.

Among 87 isolates of *E. faecalis*, 2 isolates were *vanA* positive using multiplex-PCR and duplex-LAMP assay, while MIC of 8 isolates against vancomycin were more than 32 *μ*g/mL. The results are shown in Table 4.

## 4. Discussion

*E. faecalis* is one of the most important bacterial pathogens in nosocomial infections such as surgical site, urinary tract, and bloodstream infections [18]. Vancomycin is still active against some multidrug-resistant bacteria and is therefore considered the last effective antibiotic. The vancomycin resistance *Enterococcus* (VRE), which first appeared three decades ago, is now a serious threat to public health because it has spread rapidly to many parts of the world. Therefore, rapid, sensitive, and reliable diagnosis of VRE is essential in reducing morbidity and mortality of this pathogen. The *VanA* gene is the most common phenotype observed in hospital isolates and is increasingly predominant in VRE isolates [19, 20]. Based on the results, *E. faecium* isolates showed high resistance to antibiotics compared to *E. faecalis* in our study. However, 91.66% of them were resistant to ampicillin. In contrast, ampicillin resistance was observed in only 5.81% of *E. faecalis* isolates. Several studies have reported that ampicillin resistance is very common among clinical isolates of *E. faecium* [21–23]. The results of MIC method showed that 8 isolates were phenotypically resistant to vancomycin.

The prevalence of *Enterococcus* strains by culture method in different clinical isolates including 79.63%, 16.66%, 1.85%, 0.92%, and 0.92% were reported in *E. faecalis*, *E. faecium*, *E. avium*, *E. psudoavium*, and *E. raffinosus*, respectively. Similar to our study, *E. faecalis* was reported from 80 to 90% of all enterococcal-related infections [24–26]. Sensitivity, specificity, positive predicting value, and negative predicting value, of both methods of PCR and LAMP in detecting *E. faecalis*, were 94.19%, 72.73%, 76.19%, and 93.10%. These results were approximately the same which was reported by Benadof et al. (96.8%, 76.0%, 67.7%, and 97.9%, respectively [27]). LAMP assay were recognized 87 isolates as *E. faecalis* that was in perfect agreement with multiplex-PCR assay. It means that the agreement of PCR and LAMP was 94%. Agreement of LAMP and gold standard method for detection of *E. faecalis* was %97 that was the highest rate of agreement that was reported [27, 28]. The detection of vancomycin resistance has been done using multiplex-PCR and duplex-LAMP, and the results were compared with microdilution test as a gold standard. The results were showed that 8 samples had the MIC of more than 32 *μ*g/ml but only two samples were positive for *vanA* gene using PCR and LAMP. The duplex-LAMP method was highly analytically sensitive, as DNA with as few as six target gene copies was detectable in the LAMP reaction. Amplification of the target sequence was confirmed by visualization on agarose gel electrophoresis with or without restriction digestion using *EcoRI*. The electrophoresis pattern of each single or duplex reaction of LAMP products were distinguished from each other even before restriction enzyme digestion. In this study, we demonstrated the usefulness of LAMP for detecting VRE infection in clinical specimen. We determined that the lowest amount of DNA template could yield a positive reaction. This notion is of importance when dealing with clinical specimen, especially under a condition where fast onsite diagnosis is necessary. The LOD for detection was found to be 10 fg target DNA in reaction within 40 min. This result clearly was lower than what reported from a previous study, with a LOD of 62.5 ng DNA [29]. The main reason for this difference is the presence of different inhibitors in the samples to which PCR is sensitive while LAMP is resistant [30]. Finally, compared to the PCR method, the LAMP assay optimized in this study can effectively identify the *vanA* gene with high sensitivity and specificity, which eliminates the use of an expensive specialized device and required only a simple water bath or heat blocker that was needed to perform the reaction.

The article "Rapid Detection of vanA Resistance Gene from E. faecalis Clinical Isolates Using Duplex Loop-Mediated Isothermal Amplification and Triplex PCR Assay" was published in 2022. Journal: Biomed Res Int.

## 5. Conclusion

In this study, duplex-LAMP was conducted for the first time for detection of *E*. *faecalis* and *vanA* gene simultaneously which was in perfect agreement with culture and multiplex-PCR. This method also has high sensitivity and specificity, cost-effective, and time-consuming with low LOD compared to other methods.

## Figures and Tables

**Figure 1:** (a) PCR product electrophoresis of *Enterococcus* isolates. Lane 1: 100 bp DNA ladder; lane 2: negative control; and lane 3: positive control with 305 bp product for *E. faecalis*, 195 bp product *for vanA*, and 109 bp product for *Enterococcus*. (b) LAMP electrophoresis of amplified *Enterococcus* isolates. Lane 1: 8: 50 bp DNA ladder; lane 2: single reaction for detection of *E. faecalis*; lane 3: the duplex-LAMP for detection of *E. faecalis* and *vanA* gene; lane 4: the single reaction for detection of *vanA*; lane 5: *EcoRI* digested single reaction for detection *of E. faecalis*; lane 6: *EcoRI* digested of duplex-LAMP for detection of *E. faecalis* and *vanA* gene; and lane 7: *EcoRI* digested of single reaction for detection of *vanA.*

**Figure 2:** Result of analytical specificity of the LAMP primers. (a) Positive and negative reaction of the LAMP method. Naked eyes visual detection of LAMP reaction with purified DNA of *non-E. faecalis*. 1: positive control; 2: negative control; 3: *E. faecium*; 4: *E. avium*; 5: *E. raffinosus*; 6: *E. psudoavium*; 7: *E. hirae*; 8: *E. durans*; 9: S. *pneumoniae*; and 10: *S. aureus*. (b) PCR product for analytical specificity of primers. Lane 1: 100 bp DNA ladder; lane 2: negative control; and lane 3: positive control with 109 bp product for enterococcus, 195 bp product for *vanA* gene, and 305 bp product for *E. faecalis*.

**Figure 3:** (a) LAMP primers targeting the *VanA* (*E. faecalis*) gene were used in the serial dilutions to determine limit of detection. 1: negative control; 2: positive control; 3: 1 ng; 4: 0.01 ng; 5: 1 pg; 6: 0.01 pg; 7: 1 fg (LOD of *E. faecalis*); 8: 0.1 fg; 9: 0.01 fg; 10: 1 Ag from purify DNA of *E. faecalis.* (b) LOD of *E. faecalis* by PCR assay. 1: 100 bp DNA ladder; 2: positive control (109 bp *Enterococcus*, 195 bp *vanA*, and 305 bp *E. faecalis*); 3: negative control; 4: 10 ng; 5: 1 g; 6 : 0.1 ng; 7: 10 pg (LOD of *vanA*); 8: 1 pg; 9: 0.1 pg (LOD of *E. faecalis*); 10: 10 fg (LOD of *Enterococcus*); 11: 1 fg; 12: 0.1 fg; and 13: 0.01 fg from purify DNA of *E. faecalis.*

**Table 1:** List of PCR and LAMP primers that were designed and used in this study.

Primer name	Sequence (5′ to 3′)	Product size	Reference
*Enterococcus tuf* gene	F: TAC TGA CAA ACC ATT CAT GAT G R: TTC GTC ACC AAC GCG AAC	109 bp	This study
*E. feacalis ddl* gene	F: CCA CAA GTA CCA TTC GTG C R: GCG ACA TCT TTC ACC ACT TC	305 bp	This study
Tn 1546 *VanA* gene	F: TCG TTG ACA TAC ATC GTT GC R: TGT CTT GCC GAT TCA ATT GC	195 bp	This study
*Van A* BIP	CCGCAGACCTTTCAGCAGAG-GAATTC-GAGCGCTTTATATATTTTTTTTGCC		This study
*Van A* FIP	GAACGGTTATAACTGCGTTTTCAG-GAATTC-ATCTTTCGTATTCATCAGGAAG		This study
*Van A* B3	GGGCTAGACCTCTACAGC		This study
*Van A* F3	AAATCAGGCTGCAGTACG		This study
*Van A* LB	AGCGAGGACGGATACAGGA		This study
*Van A* LF	AGCCTTTTTCCGGCTCGA		This study
*E. faecalis* BIP	CATTCCACAAGTACCATTCGTGC-GAATTC-CCTTCACATTTTTCAAAGACTTC		This study
*E. faecalis* FIP	TCCATTGCGTTAACGCTAGCTA-GAATTC-ATGGAAACCATTAATATGCCTT		This study
*E. faecalis* B3	AGGTTTAACAAAGACCGGATA		This study
*E. faecalis* F3	AGATGGAACAATTCAAGGATTC		This study
*E. faecalis* LB	TAAGAAGTGACTGGAAAGGAAATCC		This study
*E. faecalis* LF	GACACCCGCGCCTACATAA		This study

The article "Rapid Detection of vanA Resistance Gene from E. faecalis Clinical Isolates Using Duplex Loop-Mediated Isothermal Amplification and Triplex PCR Assay" was published in 2022. Journal: Biomed Res Int.

**Table 2:** Distribution of *Enterococcus* strains isolated from different clinical samples.

Samples	*E. faecalis*	*E. faecium*	*E. avium*	*E. psudoavium*	*E. raffinosus*	Total
Urine	53	5	0	0	0	58
Blood	10	9	1	1	1	22
Wound	20	4	1	0	0	25
CSF	4	0	0	0	0	4
Total	86	18	2	1	1	108

**Table 3:** Clinical specificity and sensitivity of the PCR, LAMP, and API.

	PCR		LAMP		API	
Sensitivity	=94.19%	95% CI: 86.94% to 98.06%	=94.19%	95% CI: 86.94% to 98.06%	=93.57%	95% CI: 86.00% to 97.92%
Specificity	=72.73%	95% CI: 49.78% to 89.20%	=72.73%	95% CI: 49.78% to 89.20%	=53.57%	95% CI: 33.88% to 72.47%
Positive likelihood ratio	=3.45	95% CI: 1.74% to 6.85%	=3.45	95% CI: 1.74% to 6.85%	=2.02	95% CI: 1.35% to 3.02%
Negative likelihood ratio	=0.08	95% CI: 0.03% to 0.19%	=0.08	95% CI: 0.03% to 0.19%	=0.12	95% CI: 0.05% to 0.29%
Disease prevalence	=79.63% (∗)	95% CI: 70.80% to 86.77%	=79.63% (∗)	95% CI: 70.80% to 89.20%	=74.07% (∗)	95% CI: 64.75% to 82.03%
Positive predictive value	=93.10% (∗)	95% CI: 85.58% to 97.41%	=93.10% (∗)	95% CI: 85.58% to 97.41%	=85.23% (∗)	95% CI: 76.06% to 91.89%
Negative predictive value	=76.19% (∗)	95% CI: 52.83% to 91.69%	=76.19% (∗)	95% CI: 52.83% to 91.69%	=75.00% (∗)	95% CI: 50.89% to 91.25%
KAPA	0.8981		0.8981		0.8333	

**Table 4:** Detection of *vanA* gene using PCR and LAMP in comparison with MIC against vancomycin in *E. faecalis* isolates.

Test	Result	
	Positive	Negative
MIC	8	78
PCR *vanA*	2	84
LAMP *vanA*	2	84

## Data Availability

All the data supporting the findings are contained within the manuscript.
